# The impact of China’s digital inclusive financial development gap on the optimization of rural consumption structure

**DOI:** 10.1371/journal.pone.0308412

**Published:** 2024-08-08

**Authors:** Shuaihang Yi, Ying Qi, Yongxiang Ya, Jiaying Shi, Yiniu Cui

**Affiliations:** 1 School of Economics and Management, Yunnan Normal University, Kunming, China; 2 School of Economics, Yunnan University, Kunming, China; Zhengzhou University, CHINA

## Abstract

Implementing the rural revitalization strategy is crucial for ensuring and enhancing the livelihoods of the vast rural population. The upgrading of rural consumption reflects the gradual realization of rural residents’ pursuit of a better life, and the rapid development of digital inclusive finance provides strong support for this. Based on the Digital Inclusive Finance Index released by Peking University and panel data from 30 provinces across the country, this study examines the role of digital inclusive finance in optimizing rural consumption structure through the mediation effect model and analyzes its spatial spillover effects using the spatial Durbin model. The research shows that narrowing the development gap in digital inclusive finance is crucial for upgrading the rural consumption structure, which helps to promote rural residents’ transition to higher-level consumption. Through the analysis of the spatial Durbin model, this study finds spatial spillover effects in this process, meaning that financial development in a particular region promotes local development but inhibits development in neighboring areas. Among various dimensions, the impact of breadth of coverage is the most significant. This trend of financial development affects consumption structure by increasing agricultural productivity and rural residents’ operational income, particularly highlighting its impact on operational income. However, there are significant differences between the eastern and central-western regions in optimizing rural consumption structure, with the eastern region benefiting more while the effects in the central-western region are limited and sometimes even negative. Therefore, regional characteristics should be fully considered in policy formulation to narrow the development gap in digital inclusive finance and achieve high-quality and sustainable development.

## 1. Introduction

As China enters a new phase of its economy, the countryside is in a period of transition, urgently requiring solutions to narrow the urban-rural divide and address rural development deficiencies, aiming to achieve the grand goal of fully building a modern socialist country. The Ministry of Agriculture and Rural Affairs of China pointed out that in 2022, the per capita income ratio between urban and rural residents was 2.45. Although the rural poor population has largely been lifted out of poverty, the driving force behind rural development still needs to be continually strengthened. In light of this, the rural revitalization strategy was explicitly proposed in the report of the 19th National Congress of the Communist Party of China. This strategy is not only key to current development but also a major strategic plan of the Party in the new era [1]. The rural revitalization strategy has profound significance in addressing issues related to agriculture, rural areas, and farmers. It is considered a core driving force behind the country’s sustained economic growth and thus receives high attention from policy makers and the academic community. In the journey towards rural revitalization, rural consumption plays a vital role. As one of the three major drivers of economic growth, consumption plays a critical role in promoting economic development, advancing industrial upgrading, achieving structural adjustment, and creating job opportunities [2]. Its potential, if not fully tapped, also limits China’s economic growth to some extent. The role of rural consumption in rural revitalization should not be underestimated; it not only directly drives rural economic growth but is also key to improving the rural economic structure, enhancing the quality of life for farmers, and promoting integrated urban-rural development [3]. Therefore, deeply exploring the structure of rural consumption holds extremely important practical significance and strategic value for the modernization of the country’s agriculture and rural areas [4].

The rise of digital inclusive finance is widely considered as a key to solving the development dilemma of rural economy. In the "Opinions of the Central Committee of the Communist Party of China and the State Council on Comprehensively Promoting Rural Revitalization and Accelerating Agricultural and Rural Modernization" issued in 2021, the strategy of "promoting the development of rural digital inclusive finance" was explicitly put forward for the first time, marking the first inclusion of this concept at the national policy level. The document emphasizes that the foundation of national rejuvenation must be rooted in rural revitalization, and addressing the issues related to agriculture, rural areas, and farmers is a core focus of the Party’s work. Research on rural development has shown that the long-standing dual economic structure in rural areas has led to structural mismatches in rural credit supply and demand, which may impede liquidity and resource allocation capabilities, thereby hindering the development of local industries. Additionally, the urban-rural digital divide constrains the wealth growth of rural households, as rural areas struggle to receive sufficient financial support. Therefore, rural digital inclusive finance is seen as a key driver of advancing the rural revitalization strategy. By enhancing the universality and inclusiveness of financial services, it can promote fund mobility, financing convenience, and deepen rural consumption. According to the "2023 China Financial Stability Report" released by the People’s Bank of China, digital inclusive financial services have covered nearly 80% of the adult population, with a significant proportion being rural residents. The widespread adoption of digital financial services has brought diversity to the consumption patterns of rural residents and provided a fertile ground for the emergence and growth of non-traditional consumption models.

Although digital inclusive finance in China is rapidly advancing, there is significant imbalance in its development among different regions, posing a considerable challenge to the innovation of consumption patterns in rural areas. According to the "China Internet Development Report" (2023) released by the National Information Center, the eastern coastal regions demonstrate a significant advantage in the inclusiveness of digital inclusive finance, with a coverage rate as high as 82%, while the coverage rate in western regions is only 56%. Combining the analysis of digital inclusive finance in the previous text, this regional imbalance not only limits the release of consumption potential but may also exacerbate the economic disparities among regions. Clearly, the imbalance in the development of digital inclusive finance cannot be overlooked.

Against this backdrop, the disparity in the development of digital inclusive finance significantly impacts rural consumption [5]. While a vast body of existing research focuses on the positive effects of digital inclusive finance on rural consumption, the perspective adopted in evaluating its impact on changes in rural consumption structures has its limitations. These limitations are primarily evident in the following areas: (1) The research perspective tends to be narrow, lacking a comprehensive examination of the impact on rural consumption structures from the angle of uneven development of digital inclusive finance. (2) The analysis is relatively simplistic, missing out on an integrated and comprehensive analysis of the relationship and mechanisms between the development gap in digital inclusive finance and rural consumption structures. (3) In studies analyzing the impact of digital inclusive finance on rural consumption structures, there’s a lack of in-depth research on its spatial effects. To address these research gaps, this study proposes the following improvements and directions for development: (1) This study employs a spatial Durbin model to explore the impact of the development disparity in digital inclusive finance on rural consumption structures, thereby overcoming the methodological limitations of previous research. This approach enables a more comprehensive understanding of the relationship between the development gap in digital inclusive finance and rural consumption structures, offering new perspectives and methodological support for the formulation and implementation of rural revitalization policies. (2) This research focuses on the issue of development disparities in digital inclusive finance, exploring its impact on rural consumption structures, especially in terms of regional differences or specific sub-dimensions and overall impact mechanisms. (3) By using the spatial Durbin model, this study examines the spatial effects of the development disparity in digital inclusive finance. It aims to provide a new perspective on rural revitalization, deeply understanding the impact of digital inclusive finance in promoting the optimization of rural consumption structures, its mechanisms, and examining its spatial effects against the backdrop of insufficient and uneven development of digital inclusive finance across different regions.

## 2. Literature review and research hypotheses

### 2.1 Digital inclusive finance and rural consumption structure

For a long time, the academic community has delved into the impact of digital inclusive finance on rural revitalization from multiple perspectives, gradually recognizing its non-negligible role in stimulating rural consumption. Chen et al. (2022) conducted empirical analysis from the perspective of family entrepreneurship and found that digital inclusive finance effectively reduces the barriers for rural residents to access financial services, simplifies payment processes, enhances fund liquidity, drives rural consumption, and reduces the poverty vulnerability of Chinese rural households [6]. Furthermore, digital inclusive finance also narrows the urban-rural income gap, reduces income volatility, and accelerates digital circulation, thereby enhancing the entrepreneurial capabilities and financial accessibility of rural residents [7]. These measures indirectly increase household income and educational levels, thus driving the reform of rural consumption, promoting the integration and upgrading of rural industries, and enhancing agricultural productivity. Tian He et al. (2023) have thoroughly analyzed how digital inclusive finance optimizes the income structure of low-income rural families by diversifying livelihood resources [8]. Yu et al. (2022) found through empirical evidence that digital inclusive finance not only expands the scale of consumption but also improves the structure of consumption, especially promoting basic and luxury consumption significantly, highlighting its potential in revitalizing rural family consumption [9].

Based on this, we propose Hypothesis H1(a): The reduction in the development gap of digital inclusive finance will help to upgrade the rural consumption structure.

Inclusivity and accessibility are key features of digital inclusive finance. Due to these characteristics, digital inclusive finance can penetrate more deeply and broadly compared to traditional finance, and its developmental impact is likely not confined to the local area [10]. Considering the spatial dimension reveals the characteristic of factor mobility, which can overcome geographical transaction barriers. This phenomenon leads to an interdependent relationship in economic development among neighboring regions. In the modern financial system, digital inclusive finance, supported by extensively built infrastructure, effectively eliminates the constraints of geography and time on financial services, promoting the aggregation and dissemination of financial resources [11]. In this context, digital inclusive finance is not only a crucial force for inclusive economic growth in the local area but also affects neighboring regions, displaying a "siphon effect" or "demonstration effect" and presenting spatial externalities. Zhang et al. (2024) discovered that the key factors enhancing people’s welfare are the wide range of coverage and the intensive utilization in the various aspects of digital inclusive finance, with the latter exerting a more significant influence than the former [12]. Therefore, when assessing the impact of the development gap in digital inclusive finance, it is essential to consider its spatial spillover effect, especially exploring the differences among its various sub-dimensions in this impact.

Based on this, we propose Hypothesis H1(b): The development gap in digital inclusive finance has a spatial spillover effect on the rural consumption structure.

Extensive studies have led scholars to understand that significant variations exist in the development of digital inclusive finance among different regions [13]. For instance, in China, the progress of digital inclusive finance, which relies on a contemporary financial framework and is propelled by information technology and digitalization, is highly inconsistent due to disparities in economic development and infrastructure distribution across different areas. This imbalance in development is particularly pronounced in the urban-rural divide, closely linked to the uneven state of economic development, and displays its unique characteristics. The underlying reasons are multifaceted, involving structural factors such as levels of economic development, infrastructure conditions, education levels, policy support, and geographical location, all of which collectively influence the progression of digital inclusive finance. These regional differences ultimately lead to disparities in the development level of digital inclusive finance. Against the backdrop of promoting rural revitalization, exploring the relationship between regional disparities in the development of digital inclusive finance and rural consumption holds significant theoretical and practical importance for unlocking the potential of rural consumption and driving economic growth. Nonetheless, domestic academic exploration of this topic is still in its nascent stages. Li et al. (2023) demonstrate that differences in digital inclusive finance across provinces substantially influence the spending habits of urban and rural dwellers. These disparities could also alter consumption patterns in rural areas [14].

Based on this, we propose Hypothesis H1(c): The impact of the development gap in digital inclusive finance on the structure of rural consumption exhibits significant regional heterogeneity in China.

### 2.2 Digital inclusive finance, agricultural labor productivity and rural consumption structure

The advent of digital inclusive finance, with its inclusivity and accessibility, has significantly propelled local productivity enhancement, thereby improving the work efficiency of the regional workforce. Reflecting on the current state of rural development in China, agriculture still holds a dominant position in the industry structure of rural areas. Zhou and colleagues (2022) created a Logit model, which indicates that improving financial literacy can enhance the growth of digital inclusive finance, thereby increasing farmers’ capacity to obtain financial resources [15]. As a result, reducing the disparity in digital inclusive finance development is expected to improve agricultural productivity. According to the theory of induced technological change, rational agricultural households will increase their input of relatively abundant and cheaper production factors in substitution for those that are scarce and costly. With China’s demographic dividend gradually diminishing and agricultural labor becoming a scarce factor, the price of labor and the opportunity cost of farming are on the rise [16]. Liu et al. (2023) employed inter-provincial panel data to develop regression models, demonstrating that digital inclusive finance’s growth can beneficially influence the modern agricultural economy and the restructuring of the agricultural industry [17]. It plays a significant role in enhancing the agricultural sector’s overall productivity, broadening agricultural industrial chains, and encouraging new forms of agriculture. This contribution from digital inclusive finance has the potential to significantly boost agricultural labor productivity. With significant improvements in agricultural labor productivity, farmers can manage and operate their lands more effectively. Sadik‐Zada et al. (2021), after empirical analysis using fixed effects, mediating effects, and threshold effects models, suggests that such progress is likely to trigger a massive shift of labor from traditional farming to manufacturing and service sectors, thereby accelerating the modernization of agriculture and promoting economic development [18]. Moreover, the transformation in labor structure and the optimization and upgrading of industries also lead to an increased demand for non-agricultural products and services, such as home appliances, education, medical care, and entertainment facilities. This, in turn, promotes a synergistic effect on consumption structure. This evolution in consumption patterns not only promotes rural residents’ pursuit of a better quality of life and enjoyment but also enriches the variety of goods and services in the rural market, meets the farmers’ demands for diversified consumption, and enhances the diversity of rural economic activities [19]. Therefore, it is posited:

H2: There exists a negative correlation between the development gap in digital inclusive finance and agricultural labor productivity, which, to some extent, facilitates the optimization of the rural consumption structure.

### 2.3 Digital inclusive finance, rural residents’ operational income and rural consumption structure

The advent of digital inclusive finance and its proliferation and development have not only facilitated the structural adjustment of the agricultural industry and the rational allocation of production factors but have also improved agricultural labor efficiency, thereby triggering changes in agricultural income. Such changes are closely associated with the operational income of rural residents. Scholars such as Ge et al. (2023) have indicated in their research that digital inclusive finance primarily enhances rural household agricultural factor allocation and, consequently, rural residents’ operational income through two mechanisms: the transfer of labor out of agriculture and the circulation of land, i.e., by reducing the agricultural labor population and the cultivated area [20]. Although, for a certain period, transfer and property incomes have a more considerable marginal effect on household consumption expenditure within the income structure of farming households, carrying a "multiplier effect," long-term perspectives, such as those presented by Liu et al. (2021) through empirical research with a Panel Data model, suggest that rural residents’ family operational income significantly impacts their consumption behavior [21]. Based on Milton Friedman’s Permanent Income Hypothesis, differences in income certainty and liquidity constraints lead to variations in the motive for precautionary savings, thereby significantly affecting consumption tendencies. Sustained income growth will more effectively promote consumption tendencies. Hence, the research hypothesis H3 is formulated as follows:

H3: Narrowing the development gap in digital inclusive finance will increase rural residents’ operational income and enhance the proportion of developmental and enjoyment-oriented consumption in their total consumption.

## 3. Methodology and data

### 3.1 Model specification

#### 3.1.1 OLS panel regression model construction

To study the impact of the development gap of digital inclusive finance on rural consumption structure, the following benchmark regression model (1) is constructed:

$${lncontri}_{it}=a_{0}+\beta_{1}{ingap}_{it}+\sum \beta_{i}{control}_{it}+{ℇ}_{it}$$ (1)

In Eq (1), *lncontri*_*it*_ represents the optimization of rural residents’ consumption structure in province *i* in year *t*, while *ingap*_*it*_ denotes the core explanatory variable of this paper, which is the development gap in digital inclusive finance in province *i* in year *t*. *β*_i_*control*_*it*_ represents the control variables in the model, including urbanization rate (*urban*), level of innovation (*rd*), degree of government intervention (*goverinter*), e-commerce level (*ecom*), and the average years of education in rural areas (*edu*). *a*_0_ represents a constant term; *ε* is a random error term.

#### 3.1.2 Construction of spatial Durbin model

To measure the spatial effect of the development gap of digital inclusive finance on the upgrading of rural consumption structure, a spatial econometric model is introduced, as shown in Formula (2).

$${lncontri}_{it}=\rho \sum_{j=1}^{n}W_{ij}{lncontri}_{it}+{\beta_{1}ingap}_{it}+\theta_{1}\sum_{j=1}^{n}W_{ij}{ingap}_{it}+\lambda X_{it}+\mu_{i}+\lambda_{t}+\varepsilon_{it}$$ (2)

In Eq (2), *i* represents area, *t* denotes year; *W* is *n*×*n* order geographical distance spatial weight matrix; *ρ* is the spatial autocorrelation coefficient of the explained variable to measure the possible spatial correlation of the explained variable between regions; *β* is the regression coefficient of explanatory variables, which measures the influence of explanatory variables on explained variables in the region; *θ* is the spatial regression coefficient of explanatory variables to measure the spatial spillover effect of explanatory variables; *X*_*it*_ denotes control variables, including urbanization rate (*urban*), level of innovation (*rd*), degree of government intervention (*goverinter*), e-commerce level (*ecom*), and the average years of education in rural areas (*edu*); *μ*_*i*_ is the spatial fixed effect, *λ*_*t*_ is the time fixed effect, *ε*_*it*_ is a random error term.

#### 3.1.3 Construction of mediating effect model

This study’s hypotheses H2 and H3 posit that the development gap in digital inclusive finance impacts rural consumption structure through pathways such as the level of financial development, agricultural labor productivity, and the operational income of rural residents. To test this mechanism, the paper employs Sobel’s method to construct a mediation effect model, as specifically illustrated in Eqs (3) and (4).

$${mediating}_{it}=a_{0}+\beta_{1}{ingap}_{it}+\sum \beta_{i}{control}_{it}+{ℇ}_{it}$$ (3)

$${lncontri}_{it}=a_{0}+\beta_{1}{mediating}_{it}+\beta_{2}{ingap}_{it}+\sum \beta_{i}{control}_{it}+{ℇ}_{it}$$ (4)

In Eqs (3) and (4), *lncontri*_*it*_ represents the optimization of rural residents’ consumption structure in province *i* in year *t*, while *ingap*_*it*_ denotes the core explanatory variable of this paper, which is the development gap in digital inclusive finance in province *i* in year *t*. *β*_i_*control*_*it*_ represents the control variables in the model, including urbanization rate (*urban*), level of innovation (*rd*), degree of government intervention (*goverinter*), e-commerce level (*ecom*), and the average years of education in rural areas (*edu*). *a*_0_ represents a constant term; *ε* is a random error term. *mediating*_*it*_ represents mediating variables, including agricultural labor productivity (*agripro*) and rural resident operating income level (*lnrurin*).

### 3.2 Variable measurement

#### 3.2.1 Dependent variable

In this study, the optimization of the rural residents’ consumption structure *lncontri* is chosen as the dependent variable. It is measured by the proportion of development and enjoyment type consumption expenditures out of the total consumption expenditure, logarithmized for analysis. A higher proportion indicates a more advanced consumption structure among rural residents. The development and enjoyment type consumption expenditures referred to in this paper include expenditures on daily living goods and services, transportation and communication, education, culture and entertainment, medical care, and other goods and services. To mitigate the effects of heteroscedasticity and multiple nonlinearities, and to reduce data volatility, the variables are subjected to natural logarithm transformation.

#### 3.2.2 Core independent variable

The inter-provincial development gap in digital inclusive finance *ingap*, as the explanatory variable for this study, is measured based on the Digital Inclusive Finance Development Index of each provincial region provided by the Digital Finance Research Center of Peking University. This gap is quantified using Eq (5), which is based on said index.

$$\mathrm{ingap}=\frac{{\left({\mathrm{Digtial}‐\mathrm{Finance}}_{\mathrm{it}}-{\mathrm{Digtial}‐\mathrm{Finance}}_{t}\right)}^{2}}{{\mathrm{Digtial}‐\mathrm{Finance}}_{\mathrm{it}}*{\mathrm{Digtial}‐\mathrm{Finance}}_{t}}$$ (5)

Among them, Digital Finance_it_ represents the digital inclusive finance development index of province *i* in period *t*, and Digital Finance_t_ represents the average digital inclusive finance development index of China in period *t*.

#### 3.2.3 Mediating variable

Given the pivotal role of agricultural development within the current rural economic ecosystem and the significant impact of durable income on rural consumption over an extended timeline—where operational income constitutes the main source of durable income for many rural residents—this paper utilizes intermediary variables that include agricultural labor productivity (*agripro*) and the level of rural residents’ operational income (*lnrurin*). Agricultural labor productivity is measured by taking the logarithm of the value obtained from dividing the gross value added of the primary sector by the rural population. The level of rural residents’ operational income is quantified by logarithm zing the value of rural operational income.

#### 3.2.4 Control variable

*(1) Urbanization level (urban)*. Measured by the proportion of urban population to the total population, which indicates the convergence of population in urban areas [22]. The growth in urbanization level speeds up the urbanization process, lowers the migration threshold for rural residents, and offers more development opportunities. Populations can find livelihoods in the less expensive suburbs and towns, while also enjoying the infrastructure and social benefits brought by urbanization, effectively improving the consumption level of rural residents. Without controlling for urbanization level, the impact of the development gap in digital inclusive finance might be incorrectly attributed to urbanization levels, leading to biased research conclusions.

*(2) Level of innovation (rd)*. This is measured by the logarithm of the number of patent applications in the region, reflecting the level of technological advancement to some extent. Innovation is a source of economic growth and can promote the development of information circulation, e-commerce expansion, and the prevalence of mobile payments, potentially offering rural residents more choices and changes in consumption. Referring to the method of Cui et al. (2023), considering the level of innovation as a control variable helps to gain deeper insights into the study of the imbalanced development of digital inclusive finance on the consumption structure of rural areas [23]. This control factor can enhance the precision and credibility of the study.

*(3) Degree of government intervention (goverinter)*. This reflects the extent of government interference in the local market and support for economic development, represented by the ratio of government fiscal expenditure to local GDP. The degree of government intervention, as a "visible hand," may have a positive impact on local infrastructure, healthcare, and agricultural policy support, possibly facilitating a shift in rural consumption from basic survival needs to more diverse and advanced consumption. Therefore, referring to Razzaq et al. (2023) study as a control variable, considering the degree of government intervention may help the academic community better understand the connection between digital inclusive finance and rural consumption [24].

*(4) Development level of e-commerce* (*ecom*). This is usually the maturity of e-commerce development in a region, measured by the proportion of enterprises with e-commerce transactions. With the increasing prosperity of e-commerce, rural residents’ income may increase, and after basic needs are met, they pursue higher-level consumption, promoting a decrease in the Engel coefficient, optimizing the consumption structure. E-commerce can also promote financial innovation and improve the convenience of credit, enabling farmers to anticipate future income and optimize consumption structures. Thus, using this as a control variable can make the assessment more comprehensive [25].

*(5) Rural education level* (*edu*). Represents the educational status of rural residents in the local area, measured by the average years of education in rural areas. Referencing the control variable setting in Jiang Dongfang’s article, this variable is used as a control variable. This is because the level of education is directly related to an individual’s financial literacy and the acceptance of emerging financial tools. Rural residents with better education may use digital financial services more efficiently, thus promoting the quality and diversity of consumption patterns. Considering the rural education level variable in research is crucial for accurately assessing the direct impact of digital inclusive finance on the rural consumption structure, which helps ensure the precision and reliability of the research findings [26].

### 3.3 Data sources

The paper selects panel data of 30 provinces in China from 2012 to 2021 (the data of Xizang region was deleted due to the lack of some data) as samples. The first data source is China Statistical Yearbook, China Rural Statistical Yearbook, Statistical Report on the Development of Internet in China, data published on the official website of the National Bureau of Statistics, the websites of provincial (district, city) statistical bureaus, and statistical bulletins published by the government over the years. The second is the "Peking University Digital Inclusive Finance Index (2012–2021)" compiled by the research team of the Peking University Digital Finance Research Center, which includes three dimensions: coverage breadth, usage depth, and degree of digitization.

### 3.4 Descriptive statistics

In the analysis of panel data from 30 provinces between 2012 and 2021, on one hand, to maintain data integrity, data related to Tibet was specifically excluded; on the other hand, to minimize data fluctuations and avoid heteroscedasticity and multiple nonlinear effects, logarithmic transformations were applied to several variables, including the rural consumption structure, rural residents’ operational income, and the level of innovation. It was observed that variations exist not only in the development gaps of digital inclusive finance across different regions but also in urbanization rates, levels of innovation, degrees of government intervention, development levels of e-commerce, and rural education levels, often exhibiting some degree of fluctuation. Descriptive statistics for the specific variables are presented in Table 1.

**Table 1:** Descriptive statistics.

Variable	Obs	Mean	SD	Min	Max
lncontri	300	3.868	0.088	3.611	4.054
ingap	300	0.014	0.027	0	0.238
agripro	300	1.164	0.550	0.361	3.231
lnrurin	300	8.416	0.401	7.155	9.226
urban	300	0.602	0.118	0.363	0.896
rd	300	9.705	1.364	5.697	12.399
goverinter	300	0.251	0.103	0.107	0.643
ecom	300	8.197	3.991	0.760	23.500
edu	300	7.813	0.602	5.848	9.741

## 4. Results and discussion

### 4.1 Data stability test

This paper conducts tests for data stationarity, including unit root tests and panel cointegration tests. The tests indicate: (1) As shown in Table 2, all variables passed at least two unit root tests, specifically FISHER, LLC, and HADRI, indicating the selected variables are appropriate; (2) The cointegration tests displayed at the end of Table 2 clearly show that the panel data met the criteria of the Westerlund cointegration test. This indicates a stable, long-term equilibrium among the variables, thereby permitting baseline and mediation effect regression analyses [27].

**Table 2:** Data stability test.

Unit root test		ingap	lncontri		agripro		lnrurin	urban
FISHER	Inverse chi-squared	188.90***	81.258		34.964		46.078	101.628***
	Inverse norma	-0.121	4.977		3.860		4.512	6.385
	Inverse logit t	-3.796***	3.843		4.239		4.885	4.686
	Modified inv	11.767***	1.941		-2.286		-1.270	3.800***
	chi-squared							
LLC	Adjusted t	-34.486***	-8.050***		-4.324***		-7.042***	-4.441***
HADRI	z	10.512***	6.932***		8.483***		8.176***	8.372***
Unit root test		rd		goverinter		ecom		edu
FISHER	Inverse chi-squared	179.681***		108.348***		239.658***		183.223***
	Inverse norma	-0.704		0.219		-5.338***		0.315
	Inverse logit t	-4.021***		-0.896		-9.884***		-4.107***
	Modified inv	10.925***		4.414***		16.401***		11.248***
	chi-squared							
LLC	Adjusted t	-9.371***		-5.906***		-16.190***		-12.575***
HADRI	z	6.302***		7.077***		7.893***		4.902***
panel cointegration tests		statistic		p-value				
Westerlund		6.016		0.0000				

Standard errors in parentheses

* p<0.1

** p<0.05

*** p<0.01.

### 4.2 benchmark regression

In this paper, Table 3 displays the baseline regression outcomes. More precisely, the first column details the regression findings excluding extra control variables, focusing on the digital financial inclusion gap as the explanatory factor and the rural consumption structure as the outcome variable. Columns (2) to (6) sequentially add control variables such as urbanization rate, government intervention, e-commerce development, rural education level, and innovation level. As more variables are introduced into the model, an improvement in the model’s fit can be observed, indicating that the selected key explanatory variables and control variables are more appropriate. Furthermore, the digital financial inclusion gap is highly significant at the 1% level, significantly affecting the optimization of rural consumption structure. This supports hypothesis H1(a).

**Table 3:** OLS regression.

	lncontri					
	(1)	(2)	(3)	(4)	(5)	(6)
ingap	-1.029*** (0.179)	-0.73*** (0.18)	-0.877*** (0.182)	-0.93*** (0.183)	-0.998*** (0.183)	-1.036*** (0.181)
urban		-.225*** (0.041)	-0.164*** (0.044)	-0.127** (0.049)	-0.047 (0.056)	-0.083 (0.057)
goverinter			0.166*** (0.049)	0.173*** (0.049)	0.12** (0.052)	0.288*** (0.076)
ecom				-0.002* (0.001)	-0.002* (0.001)	-0.004*** (0.001)
edu					-0.029*** (0.01)	-0.024** (0.010)
rd						0.018 (0.006)
Constant	3.882*** (0.005)	4.013*** (0.025)	3.937*** (0.033)	3.932*** (0.033)	4.126*** (0.077)	3.911*** (0.105)
Observersions	300	300	300	300	300	300
provinces	30	30	30	30	30	30

Standard errors in parentheses

* p<0.1

** p<0.05

*** p<0.01.

Specifically, for every one percentage point reduction in the digital financial inclusion gap, there is an average increase of 1.036 percentage points in the optimization of rural consumption structure. This change in digital financial inclusion can significantly stimulate the consumption potential of rural households, having a more pronounced effect on the promotion of developmental and enjoyment-type consumption. Since developmental and enjoyment-type consumption represents an upgrade in consumption structure, it means that digital financial inclusion significantly promotes the optimization of residential consumption structure. In the regression results, the level of government intervention and innovation have a positive effect on optimizing the rural consumption structure, suggesting that areas with strong government support and high technological levels have higher household incomes and better quality of life, which in turn stimulates consumption. The quality of education in rural areas and the growth of e-commerce appear to hinder the improvement of the consumption patterns in these regions. This could stem from the irregular impacts observed in the advancement of rural education and e-commerce. Moreover, the rate of urbanization diminishes the influence of the disparity in digital financial inclusion on refining the consumption structure in rural areas. An analysis of the control variable coefficients reveals that the effects of both urbanization rate and level of innovation are negligible.

### 4.3 Spatial Durbin regression

#### 4.3.1 Moran index test

When deciding whether to use a spatial econometric model for analyzing a study, a crucial step is to verify the presence of spatial autocorrelation in the data. This requires utilizing Moran’s I index to test the spatial correlation of both the digital financial inclusion gap and the rural consumption structure. Table 4, based on a spatial matrix constructed from geographic distance matrices, shows that from 2012 to 2021, the Moran’s I indices for rural consumption structure and the digital financial inclusion gap index were significant at the 5% or 10% level, except for the rural consumption structure in 2021 and the digital financial inclusion gap in 2016.

**Table 4:** Moran I test results.

Year	lncontri	ingap
2012	0.135* (0.095)	0.158** (0.090)
2013	0.156** (0.096)	0.132* (0.090)
2014	0.129* (0.095)	0.148** (0.087)
2015	0.137* (0.095)	0.153** (0.085)
2016	0.191** (0.096)	0.101 (0.085)
2017	0.140* (0.094)	0.138** (0.085)
2018	0.131* (0.094)	0.159** (0.086)
2019	0.149** (0.093)	0.158** (0.085)
2020	0.154** (0.096)	0.159** (0.085)
2021	0.116 (0.096)	0.166** (0.085)

Standard errors in parentheses

* p<0.1

** p<0.05

*** p<0.01.

Fig 1 presents the Moran scatterplot for the digital financial inclusion gap in 2012, 1(a), revealing that 17 provinces (accounting for 56.67%) are located in the third quadrant, and similarly, the Moran scatterplot for the digital financial inclusion gap in 2021, 1(b), shows that 13 provinces (43.33%) are in the third quadrant, indicating a low-low clustering characteristic, which suggests positive spatial autocorrelation for this indicator. Likewise, the Moran scatterplot for the rural consumption structure in 2012, 1(c), indicates that 10 provinces (33.33%) are located in the first quadrant, and 9 provinces (30.00%) are in the third quadrant. According to the Moran scatterplot for the rural consumption structure in 2021, 1(d), 10 provinces (33.33%) are in the first quadrant, and 8 provinces (26.67%) are in the third quadrant, showing characteristics of both high-high and low-low clustering, which also indicates positive spatial autocorrelation for this index.

**Fig 1:** Moran’s I scatter plot in2012 and 2021. (a) Moran scatter plot of the development gap in digital inclusive finance in 2012, (b) Moran scatter plot of the development gap in digital inclusive finance in 2021, (c) Moran scatter plot of rural consumption structure in 2012, (d) Moran scatter plot of rural consumption structure in 2021.

#### 4.3.2 Spatial Durbin regression

In this investigation, the spatial Durbin model was employed to examine the regional spillover effects of the digital financial inclusion gap on optimizing rural consumption structure. Prior to performing the spatial Durbin regression analysis, preliminary tests were conducted. The results from Table 5 led to the selection of the most suitable spatial regression model using Wald and LR tests, both significant at the 1% level. Consequently, the spatial Durbin models could not be simplified to SEM or SAR models, reinforcing its appropriateness for this analysis. The choice between a random effects model and a fixed effects model was made via the Hausman test, which, at the 1% significance level, favored the fixed effects model. Therefore, the study ultimately utilized a fixed effects spatial Durbin model to assess the impact of digital finance on employment structure. Further comparison between time effects and individual effects showed that the double fixed effects model was preferable. Significant regression coefficients at the 1% level were 68.320 for the individual effects and 547.950 for the time effects, both indicating substantial impacts.

**Table 5:** Spatial regression model validation.

LR_ind	68.320***
LR_time	547.950***
Hausman	63.950***
Wald_error	43.280***
Wald_lag	43.660***
Log-likelihood	684.856
LR_error	40.730***
LR_lag	40.750***

Standard errors in parentheses; * p<0.1, ** p<0.05

*** p<0.01.

The data in Table 6 clearly reveals that the digital financial inclusion gap (*ingap*) has a significant positive impact on the upgrading of rural consumption structures. The coefficient for (Main) is shown as -0.218 and is significant at the 5% level. This effect not only significantly optimizes the rural consumption structure within provinces but also spreads to neighboring provinces, creating a spillover effect that has a suppressive impact on the upgrading of rural consumption structures in adjacent areas. According to Table 6 (Mx), the narrowing of the digital financial inclusion gap shows a significant spatial spillover effect on the optimization of rural consumption structures at the 1% level, with a coefficient of 0.781. This demonstrates that the impact of the digital financial inclusion gap on rural consumption structures is consistent with previous findings, thereby validating hypothesis H1(b).

**Table 6:** Spatial regression results.

	Main	WX
ingap	-0.218** (0.105)	0.781*** (0.259)
urban	0.059 (0.147)	-0.646** (0.278)
goverinter	-0.083 (0.083)	-0.244 (0.163)
ecom	0.001 (0.001)	-0.004* (0.002)
edu	-0.012 (0.010)	0.066** (0.026)
rd	-1.462 (1.162)	-10.543*** (2.659)
sigma2_e	0.001*** (0.000)	
Observersions	300	
provinces	30	

Standard errors in parentheses; * p<0.1

** p<0.05

*** p<0.01.

Why, then, do the direct effects and spatial spillover effects show opposite results? One possible explanation is the phenomenon known as the "siphoning effect" when examining the regional dynamics of digital financial inclusion. Specifically, when a region’s digital financial inclusion gap is smaller than its surrounding areas, it is better able to perform resource allocation functions, attracting various types of resources from nearby areas, such as human capital and natural resources, to flow into itself. The digital financial inclusion gap reflects the uneven characteristics of digital financial inclusion between regions. Observing the prevalence and depth of digital financial services across different regions shows a clear gradient of decline, from economically developed areas to relatively backward areas. In this process, the latter significantly lacks the breadth and quality of digital infrastructure compared to the former, indicating that regions with later development find it difficult to enjoy the economic growth benefits brought by digital financial inclusion. Furthermore, the market order for digital financial inclusion has not yet fully formed, and the rules between different regions face friction [28]. This situation further exacerbates the uneven distribution of resources, leading to resources flowing from areas lacking financial services to those that are already wealthy, have higher production efficiency, and offer more lucrative investment returns, intensifying the so-called "siphoning effect".

This paper delves into the effects of regional rural consumption patterns by analyzing and contrasting the disparities in coverage breadth (*BOCgap*), usage depth (*DEPgap*), and digitalization level (*DODgap*) within digital financial inclusion frameworks. It aims to pinpoint how various facets of digital financial inclusion influence rural spending behaviors. By evaluating digital financial inclusion’s multiple dimensions, the study highlights the importance of coverage breadth as a crucial metric for gauging digital finance inclusivity, which is vital for gauging its advancement. The emergence of technologies such as the internet, big data, and blockchain has greatly enhanced the accessibility and convenience of financial services for communities previously excluded, particularly affecting rural consumption dynamics. The usage depth metric of digital financial inclusion indicates the adoption rate of diverse credit offerings, essential for fueling local consumption growth; while the digitalization degree showcases the practical convenience and financial advantages of digital financial tools. According to the spatial heterogeneity regression outcomes presented in Table 7, a reduced coverage breadth disparity in column (1) fosters an upgrade in the local rural consumption framework and deters enhancement in neighboring regions’ consumption patterns. In contrast, columns (2) and (3) demonstrate that disparities in usage depth and digitalization degree significantly impact the overall rural consumption structure through a notable spatial spillover effect.

**Table 7:** Regression results of spatial heterogeneity across different dimensions.

	(1) BOCgap		(2) DEPgap		(3) DODgap	
	Main	WX	Main	WX	Main	WX
BOCgap	-0.217*** (0.054)	0.500*** (0.148)				
DEPgap			0.023 (0.044)	0.247*** (0.095)		
DODgap					0.306 (0.310)	-1.537** (0.781)
urban	0.179 (0.148)	-0.893***	0.036 (0.143)	-0.404 (0.284)	0.149 (0.146)	-0.752*** (0.289)
goverinter	-0.081 (0.082)	-0.229 (0.161)	-0.095 (0.082)	-0.175 (0.161)	-0.076 (0.085)	-0.242 (0.166)
ecom	-0.000 (0.001)	-0.001 (0.003)	0.001 (0.001)	-0.006*** (0.002)	0.002 (0.001)	-0.006*** (0.002)
edu	-0.007 (0.001)	0.004* (0.025)	-0.008 (0.011)	0.067** (0.256)	-0.003 (0.011)	0.065** (0.026)
rd	-1.526 (1.143)	-9.506*** (2.620)	-1.646 (1.166)	-11.428*** (2.671)	-1.994* (1.192)	-9.703*** (2.719)
sigma2_e	0.001*** (0.000)		0.001*** (0.000)		0.001*** (0.000)	
Observersions	300		300		300	
provinces	30		30		30	

Standard errors in parentheses

* p<0.1

** p<0.05

*** p<0.01.

The emergence of this phenomenon is attributed to the narrowing of the breadth of coverage gap, which allows surrounding markets to connect through digital finance, becoming a unified whole. This integration generates increased product demand, thereby fostering rural consumption in neighboring areas and extending inclusive financial services to a broader rural region, enabling more rural residents to enjoy the conveniences offered by inclusive finance and enhancing financial efficiency. The lack of significant impact from the depth of usage gap might be due to the broad coverage of digital inclusive finance, yet insufficient depth of use in some areas, which does not significantly contribute to income convergence, thereby not significantly affecting rural consumption. Meanwhile, with the rapid expansion of the "Village to Village" highway network, rural areas’ ability to access financial resources is no longer severely constrained by geographical distances [29]. Currently, the primary obstacle to rural financial development is the lack of a diversified supply of financial services. Therefore, in advancing the integration process of urban and rural areas, the role that the level of digitalization in digital inclusive finance can play remains limited, especially as indicated in Table 7 (3), where the negative WX coefficient suggests that digitalization helps to alleviate information asymmetry, narrowing the "digital divide" in rural areas. This allows products from the local region to flow more conveniently to other areas’ markets, aiding in the optimization of consumption structures in neighboring areas.

### 4.4 Robustness and endogeneity test

#### 4.4.1 Robustness test

In conducting robustness tests, the local economic development level is measured by taking the logarithm of GDP from different provinces, resulting in *lnGDP* and the local internet development level is represented by the number of mobile phone users per hundred people, denoted as web. After including these two control variables, the regression results are shown in Table 8 (1) and (2). Additionally, the regression is performed with a one-period lag for both the dependent variable (*lncontri*) and the independent variable (*ingap*), with the regression coefficients in Table 8 (3) and (4) being significantly negative. These outcomes are consistent with the baseline regression results, indicating the robustness of the research findings.

**Table 8:** Robustness test of benchmark regression.

	(1)	(2)	(3)	(4)
L.ingap				-1.026*** (0.204)
ingap	-0.616*** (0.207)	-0.737*** (0.203)	-2.317*** (0.366)	
urban	0.183** (0.075)	0.001 (0.084)	-0.071 (0.71)	-0.145** (0.070)
goverinter	0.085 (0.053)	-0.005 (0.055)	0.219*** (0.059)	0.144** (0.578)
ecom	-0.003** (0.001)	-0.005*** (0.001)	-0.005*** (0.002)	-0.005*** (0.002)
edu	-0.022** (0.01)	-0.033*** (0.01)	-0.034*** (0.011)	-0.034*** (0.011)
rd	2.32*** (0.769)	2.127*** (0.748)	2.453*** (0.897)	1.801** (0.865)
lnGDP	-0.136*** (0.022)	-0.137*** (0.021)		
web		0.002*** (0.000)		
Constant	5.165*** (0.179)	5.257*** (0.175)	4.145*** (0.086)	4.218*** (0.086)
Observersions	300	300	270	270
provinces	30	30	30	30
R-squared	0.333	0.374	0.270	0.252

Standard errors in parentheses

* p<0.1

** p<0.05

*** p<0.01.

#### 4.4.2 Endogeneity test

The sections above have shown that bridging the digital financial inclusion gap has greatly improved the consumption patterns in rural areas. Nonetheless, from a theoretical standpoint, the findings of this study are still susceptible to endogeneity concerns. To bolster the findings’ credibility, this study utilizes the two-stage least squares approach, the Generalized Method of Moments (GMM), and the fixed effects model as strategies to counter potential endogeneity. These methods aim to rectify the issues of endogeneity in regression analyses. According to the results displayed in Table 9, employing these three analytical techniques confirms that the initial hypothesis of the study remains valid, ensuring that the research outcomes are dependable even after conducting tests for endogeneity.

**Table 9:** Endogeneity test.

	(1)2sls	(2) GMM	(3) Fix Model
L.Lncontri		0.238*** (0.039)	
ingap	-3.009*** (0.661)	-2.286*** (0 .614)	-1.119*** (0.200)
urban	-0.153* (0.079)	0.660*** (0.123)	-0.092 (0.064)
goverinter	0.213*** (0.066)	0.161*** (0.060)	0.146*** (0.054)
ecom	-0.007*** (0.002)	-0.003** (0.001)	-0.003** (0.001)
edu	-0.035*** (0.011)	-0.008 (0.013)	-0.032*** (0.011)
rd	3.697*** (1.013)	-11.541*** (1.084)	1.093 (0.780)
Constant	4.215 (0.088)		4.162*** (0.080)
Observersions	240	240	300
provinces	30	30	20

Standard errors in parentheses

* p<0.1

** p<0.05

*** p<0.01.

To ensure the reliability of the GMM model results, some necessary tests need to be conducted. Table 10 reports the results, which indicate that there is no autocorrelation of order two in the random disturbances according to the p-value of AR(1). The Sargan test result shows that there is no problem of overidentification of instrumental variables, indicating that the estimation results are valid.

**Table 10:** GMM model test.

	AR(1)	AR(2)	Sargan
GMM	-3.32***	-0.34	176.16***

Standard errors in parentheses; * p<0.1, ** p<0.05

*** p<0.01.

### 4.5 Regional heterogeneity analysis

The gap in the development of digital inclusive finance originates from differences between regions, influenced by factors including economic development, industrial structure, population demographics, government intervention, and income levels. These factors determine the varying impacts of this financial development gap on rural consumption across the eastern, central, and western regions of the country. Observations from Table 11 reveal that the digital financial inclusion development gap significantly affects the rural consumption structure in the eastern regions, whereas in the central and western regions, it does not significantly impact rural consumption and may even hinder the optimization of consumption structure. This finding validates Hypothesis 1(c) of this study.

**Table 11:** Regional heterogeneity.

	East	Middle	West
ingap	-0.992*** (0.247)	1.771 (1.444)	0.129 (0.277)
urban	-0.369*** (0.086)	0.907*** (0.128)	-0.042 (0.135)
goverinter	0.212 (0.199)	-0.412** (0.157)	-0.141 (0.133)
ecom	-0.006*** (0.002)	-0.007** (0.003)	0.008*** (0.003)
edu	0.037* (0.022)	-0.017 (0.019)	-0.028 (0.019)
rd	0.045*** (0.009)	0.008 (0.009)	-0.015 (0.012)
Constant	3.334*** (0.152)	3.576*** (0.192)	4.250*** (0.205)
Observersions	120	90	80
R-squared	0.404	0.415	0.197

Standard errors in parentheses

* p<0.1

** p<0.05

*** p<0.01.

Typically, rural areas with lower consumption levels have weaker demand for digital financial services. In contrast, rural residents in the eastern regions have higher consumption needs, which in turn creates a stronger demand for accessibility to and services of digital inclusive finance. Due to higher levels of economic development, per capita income, and consumption levels, residents in the eastern regions are more likely to access and understand information related to digital financial services. The digital economy is also more integrated with the local industrial structure in these areas, which benefits the promotion of new consumption patterns and products and facilitates consumption upgrades. Residents in the eastern regions are more sensitive to disparities in the development of digital inclusive finance, prompting financial institutions and local governments to enhance the construction and development level of local digital financial services. This situation exacerbates the disparity in digital financial development between the eastern, central, and western regions to some extent. Conversely, the residents in the central and western regions have relatively limited purchasing power and demand, and their pace of optimizing and upgrading consumption structures is not as advanced as that in the eastern regions. Even if the gap in digital financial development is not significant in these areas, they may still face risks of over-reliance on financial services and debt. For example, in the western regions, due to lower levels of regulation and insufficient development of digital inclusive finance, the effective allocation of market resources is hampered, which not only fails to promote healthy consumption but also impedes the optimization of the consumption structure.

To delve deeper into the effects of the digital financial inclusion gap on rural spending patterns, this study develops variables to capture the coverage breadth gap, usage depth gap, and digitalization level gap. It aims to assess how disparities in these areas influence the structure of rural consumption. Detailed regression findings are presented in Table 12. Analysis of data from columns (1) to (3) of Table 12 reveals that the coefficients for coverage breadth, usage depth, and digitalization level are -0.626, -0.308, and -1.337, respectively, indicating significance at the 1% and 10% confidence intervals. This evidence points to the substantial positive impact of enhancing coverage area, usage frequency, and digitalization quality on the improvement of rural inhabitants’ consumption patterns. Notably, advancements in digitalization have the most pronounced effect on altering rural consumption behaviors, highlighting its potentially greater importance over coverage and usage metrics.

**Table 12:** Regression results of heterogeneity in various dimensions of digital inclusive finance.

	(1)	(2)	(3)
BOCgap	-0.626*** (0.102)		
DEPgap		-0.308*** (0.091)	
DODgap			-1.337* (0.731)
urban	-0.141** (0.064)	-0.105 (0.067)	-0.122* (0.067)
goverinter	0.128** (0.053)	-0.116** (0.057)	-0.067 (0.055)
ecom	-0.004*** (0.001)	-0.002 (0.001)	-0.001 (0.001)
edu	0.029*** (0.010)	-0.030*** (0.011)	-0.020* (0.011)
rd	1.371* (0.787)	0.064 (0.775)	-0.650 (0.747)
Constant	4.167*** (0.080)	4.159*** (0.084)	4.107*** (0.084)
Observersions	300	300	300
R-squared	0.262	0.199	0.177

Standard errors in parentheses

* p<0.1

** p<0.05

*** p<0.01.

### 4.6 Regression results and analysis of mediating effect model

#### 4.6.1 Mediating effect test

This research applies regression analysis with a mediation effect model to explore how agricultural labor productivity and the operational income of rural inhabitants mediate the influence of the digital financial inclusion development gap on the structure of rural consumption. The study adopts a bootstrapping approach with 500 repetitions to ascertain mediation effects. According to Table 13, _bs_1 denotes the indirect effect, and _bs_2 signifies the direct effect. Findings reveal that the _bs_1 coefficient pertaining to agricultural labor productivity stands at -0.162, indicating significance at the 10% level; additionally, the coefficient for _bs_1 linked to the operational income of rural residents is -0.453, demonstrating significance at the 1% level. This evidence supports the mediating roles of agricultural labor productivity and the operational income of rural residents in shaping the rural consumption structure. The gap in digital financial inclusion development contributes to the evolution of the rural consumption structure, with a marked mediating effect. The Sobel-Goodman test outcomes from Table 13 further corroborate the significant mediating effects of agricultural labor productivity and rural residents’ operational income.

**Table 13:** Results of mediating effect test.

	Agripro	lnrurin
Sobel	-0.162** (0.075)	-0.453*** (0.108)
Aroian	-0.162** (0.075)	-0.453*** (0.108)
Goodman	-0.162** (0.074)	-0.453*** (0.107)
_bs_1	-0.162* (0.092)	-0.453*** (0.135)
_bs_2	-0.874*** (0.267)	-0.583** (0.229)

Standard errors in parentheses

* p<0.1

** p<0.05

*** p<0.01.

#### 4.6.2 Agricultural labor productivity

Based on the findings presented in Table 14, the data in column (2) indicates a significant effect of the digital financial inclusion disparity on agricultural labor productivity, evidenced by a negative correlation at the 1% significance level. This suggests that narrowing the digital financial inclusion gap is beneficial for improving agricultural labor productivity, likely because the reduction in the digital financial inclusion gap increases loan accessibility. This enhances financial accessibility for households and individuals, alleviates credit constraints, and allows more resources to be directed towards agricultural production. Simultaneously, leveraging digital platforms facilitates financial product innovation in farmland loans, mitigates the issue of asymmetric credit information in rural areas, and precisely supports every aspect of agricultural production through digital technology. This aids farmers in improving their production and business operations and promotes continuous innovation in agricultural technology. Column (3) indicates that the development gap in digital financial inclusion and agricultural labor productivity significantly impact the optimization of rural consumption structure at the 1% level. An increase in agricultural labor productivity is likely to enhance the economic and production efficiency in rural areas, stimulate growth in rural income and the development of productive services in rural areas, improve the rural consumption environment, and encourage farmers to increase investments in production, employment, education, and other areas [30]. This enhances the consumption capacity and willingness of rural residents, subsequently optimizing the rural consumption structure. This demonstrates that agricultural labor productivity plays a partial mediating role in the influence of the digital financial inclusion development gap on the rural consumption structure, confirming the research hypothesis H2.

**Table 14:** Results of mediating effect regression analysis.

	(1) lncontri	(2) agripro	(3) lncontri
agripro			0.020** (0.009)
ingap	-1.036*** (0.181)	-7.945*** (1.180)	-0.874*** (0.193)
urban	-0.083 (0.057)	1.328*** (0.369)	-0.110* (0.058)
goverinter	0.288*** (0.076)	-0.934* (0.496)	0.307*** (0.076)
ecom	-0.004*** (0.001)	0.021** (0.009)	-0.005*** (0.001)
edu	-0.024** (0.010)	-0.060 (0.068)	-0.023** (0.010)
rd	0.018 (0.006)	-0.153*** (0.039)	0.021*** (0.006)
Constant	3.911*** (0.105)	2.495*** (0.681)	3.860*** (0.106)
Observersions	300	300	300
provinces	30	30	30

Standard errors in parentheses

* p<0.1

** p<0.05

*** p<0.01.

#### 4.6.3 Operating income of rural residents

As indicated in Table 15, the empirical results in column (1) show that the development gap in digital inclusive finance has an estimated coefficient of -1.036 on the operational income of rural residents, significantly negative. From the results in column (2), it can be seen that the regression coefficient reaches -7.580, also significantly negative. This may be because the narrowing of the digital financial inclusion gap has adjusted and optimized the allocation of agricultural production factors among rural residents. It also lowers the barriers to financing, especially for smaller-scale enterprises, which is particularly evident in rural markets dominated by micro and small enterprises, thereby significantly enhancing the operational income of rural residents. The results in column (3) reveal that the regression coefficient for the development gap in digital inclusive finance is -0.583, while the regression coefficient for rural residents’ operational income reaches 0.060, with both results being significant. Notably, rural residents’ operational income represents a continuous gain, and rural consumers show high sensitivity to fluctuations in household operational income. Observing its coefficient, rural residents’ operational income plays a mediating role, indicating that the reduction in the digital financial inclusion gap can improve rural residents’ operational income, thereby increasing their expenditure on developmental and enjoyment-related consumption [31]. In the long term, such changes in income have profound implications on the rural consumption structure. The operational income of rural residents partially mediates the effect of the digital financial inclusion development gap on the rural consumption structure, thereby validating the research hypothesis H3.

**Table 15:** Results of mediating effect regression analysis.

	(1) lncontri	(2) lnrurin	(3) lncontri
lnrurin			0.060*** (0.013)
ingap	-1.036*** (0.181)	-7.580*** (0.801)	- 0.583*** (0.200)
urban	-0.083 (0.057)	0.732*** (0.251)	-0.127** (0.056)
goverinter	0.288*** (0.076)	-1.254*** (0.336)	0.362*** (0.075)
ecom	-0.004*** (0.001)	0.002 (0.006)	-0.004*** (0.001)
edu	-0.024** (0.010)	-0.185*** (0.046)	-0.013 (0.010)
rd	0.018 (0.006)	-0.070*** (0.026)	0.022*** (0.006)
Constant	3.911*** (0.105)	10.502*** (0.462)	3.283*** (0.168)
Observersions	300	300	300
provinces	30	30	30

Standard errors in parentheses

* p<0.1

** p<0.05

*** p<0.01.

## 5. Conclusion and policy implication

### 5.1 Conclusion

Firstly, empirical results indicate that narrowing the development gap in digital financial inclusion plays a crucial role in upgrading the rural consumption structure. This not only aids in improving the rural consumption structure but also promotes the pursuit of higher-level consumption—namely developmental and enjoyment-oriented consumption—significantly increasing its proportion in total rural consumption. Additionally, digital financial inclusion exhibits a significant spatial spillover effect in promoting the upgrade of rural consumption structures. This effect manifests as digital financial inclusion being able to optimize rural consumption structures locally, while potentially limiting the optimization process in neighboring regions, a phenomenon that may be attributed to a "siphoning effect," with the breadth of coverage gap playing the most significant role in spatial effects.

Secondly, the balanced development of digital financial inclusion influences the consumption structure by improving agricultural labor productivity and increasing the operational income of rural residents, both of which play a mediating effect in this process, with the operational income of rural residents having a more significant impact.

Lastly, an examination of the development gap of digital financial inclusion across different regions of China and its varied effects across different dimensions reveals that its impact on the rural consumption structure is not constant. In eastern regions, due to more developed infrastructure and industrial structures, the narrowing of the digital financial inclusion development gap significantly promotes the optimization of consumption structures. However, in the central and western regions, due to resource scarcity and inefficient market allocation, the digital financial inclusion development gap may not significantly improve the consumption structure, and sometimes may even have a suppressive effect. Among the three dimensions of digital financial inclusion, changes in the degree of digitalization gap have a stronger driving force. Therefore, it can be concluded that there is a complex interplay between the development gap in digital financial inclusion and the optimization of rural consumption structures. This requires careful consideration of regional differences and the disparities in different dimensions of digital financial inclusion across regions when formulating relevant policies, to achieve a more balanced and sustainable development.

### 5.2 Policy implication

#### (1) Establish differentiated support to promote regional collaborative development

Given the differences among regions and the state of digital financial inclusion, governments need to perfect the layout of digital and informational infrastructure, build a digital financial support framework with distinctive regional characteristics, and dedicate efforts to the meticulous optimization of infrastructure. This includes the continuous implementation of digital rural development actions aimed at narrowing the "digital divide." This is particularly crucial for the central and western regions, where there is an urgent need to improve broadband and mobile internet coverage. Additionally, targeted educational programs should be initiated, with regular financial knowledge training sessions, especially focusing on enhancing the digital literacy and financial support for the elderly and youth. The government should fully leverage its "visible hand" by increasing government investment, implementing subsidies, and tax incentive measures to improve, thereby facilitating the proliferation of digital payment tools in rural areas and providing a sufficient prerequisite for narrowing the development gap in digital financial inclusion.

To mitigate the spatial spillover effects of digital financial inclusion, it is recommended to plan a comprehensive strategy for regional collaborative development, creating a cross-regional rural consumption collaboration platform. Infrastructure development should not only focus on upgrading local infrastructure but also on strengthening inter-regional infrastructure connectivity projects. This includes not just traditional transportation and communication infrastructure projects but also facilitating support between digital financial platforms and promoting financial knowledge education and circulation, thereby comprehensively raising the financial awareness of rural residents, and promoting balanced economic growth.

#### (2) Strengthen financial service networks and innovate product services

Optimizing the rural financial service system is an urgent priority. It’s essential to refine monetary policy support for credit institutions centered around counties, strengthen specialized service mechanisms of large banks in the "agriculture, rural areas, and farmers" sector, and clarify the support direction of rural small financial institutions for agriculture and small businesses. By province, orderly progress should be made in reforming and managing risks for rural credit cooperatives. It’s advisable to increase mobile and self-service banks in rural areas of central and western regions to ensure comprehensive coverage of financial services. Meanwhile, fully leveraging the postal savings bank network to provide basic financial services such as remittances, payments, and insurance, and strengthening cooperation with other financial institutions to expand the range of services is crucial.

Financial institutions need to closely align with the actual demands of rural areas, innovating financial products and services, especially credit service models in key sectors like food security and seed industry development. Push for the development of digital financial inclusion in rural areas and accelerate the construction of a rural credit system. Utilize resources such as the national agricultural credit guarantee system and government investment funds to enhance coordination between finance and fiscal policies, implementing loan subsidy pilot projects in agricultural areas like high-standard farmland construction and facility agriculture. For example, launching credit products combined with "Internet + Agriculture", weather index insurance, and constructing e-commerce platforms to offer pre-sale and supply chain financial solutions for agricultural products, thereby increasing farmers’ income and market competitiveness of agricultural products, effectively meeting the financial needs of rural residents, and narrowing the development gap in digital financial inclusion.

#### (3) Promote rural industrial upgrading and enhance the sustainable income of rural residents

To alleviate the economic pressures on small and marginal farmers, microloans and small-credit services should be utilized for their low barrier to entry, enabling these farmers to invest in advanced agricultural technologies and equipment. This will further enhance the efficiency and quality of agricultural output. Digital financial inclusion, integrated with blockchain and Internet of Things (IoT) technologies, can ensure the transparency and traceability of the agricultural supply chain, thereby enhancing the market competitiveness of agricultural products. Additionally, while providing funds, digital financial inclusion can also leverage its advantages in information digitization, inspiring vitality in agricultural enterprises for technological innovation and business model innovation. This promotes the development of smart agriculture, ecological agriculture, and circular agriculture, thereby overall enhancing agricultural labor productivity.

In building a modern agricultural management system, digital financial platforms offer diversified financing channels like equity crowdfunding and debt financing to agricultural enterprises, providing viable solutions for meeting the capital needs of the agricultural industry chain. Digital financial inclusion services should deepen the use of data analysis to provide agricultural operators with accurate market trend predictions and personalized business strategies, assisting them in making more scientific decisions. In the process of promoting industrial upgrading and integration, digital financial inclusion can support the integration of agriculture with other sectors like the service and tourism industries through financial support, achieving synergistic growth and value chain expansion across industries, and promoting diversified development and industrial chain upgrading in agriculture. This process can enhance the operational income of rural residents primarily engaged in agriculture. The improvement of this sustainable income will clear obstacles for narrowing the development gap in digital financial inclusion and optimizing the rural consumption structure.

## 6. Research limitations and prospects

Although this research provides many valuable insights, there are still some limitations. Firstly, the digital inclusive finance index and panel data used in this study cover 30 provincial-level administrative regions nationwide, but due to data acquisition restrictions, Tibet is not included, which may affect the representativeness of the research results nationwide. Secondly, this paper mainly focuses on the development gap of digital inclusive finance between different provinces and the national level, that is, the regional gap, and is limited by length to further explore the impact of regional differences within regions. Finally, this study found significant differences in the impact of digital inclusive finance in different regions, especially showing imbalanced effects between eastern and central-western regions. Future research should further explore the underlying reasons for this regional difference, considering various factors including infrastructure, education level, and policy environment, in order to propose more accurate regional policy recommendations and effectively narrow the development gap of digital inclusive finance.

There are several key directions worth further exploration in future research. Firstly, addressing the lack of data in the Tibet region, future research should strive to obtain and integrate more data on digital inclusive finance in Tibet to ensure the universality and representativeness of research results nationwide. This not only helps improve the current research model but also provides policymakers with more comprehensive reference. Secondly, future research should delve into the development gap of digital inclusive finance within provinces. By using more detailed data, such as hierarchical data of urban and rural areas, it can reveal the imbalanced development of digital inclusive finance within regions. This can help understand the digital divide within different regions and provide targeted solutions to narrow these gaps. In addition, future research should focus on the dynamic process of digital inclusive finance development, using time series analysis methods to explore the changing trends and development paths of digital inclusive finance at different time points. This can help identify which policies and measures have a significant impact on the development of digital inclusive finance at different stages. Another important research direction is to deeply analyze the underlying reasons for the imbalanced development of digital inclusive finance in eastern and central-western regions. Future research can use multilevel regression analysis or structural equation models, considering the interaction of multiple factors such as infrastructure construction, education level, policy environment, and economic development, to explore how these factors jointly affect the development of digital inclusive finance. Finally, future research should pay more attention to the comprehensive impact of digital inclusive finance on socio-economic development, including its impact on income distribution, fair education, medical services, and other aspects. By constructing a comprehensive evaluation system, a more comprehensive assessment of the social benefits of digital inclusive finance can be made, providing a scientific basis for formulating a more comprehensive strategy for the development of digital inclusive finance. These future research directions can not only deepen the understanding of digital inclusive finance but also provide policymakers with more accurate and effective policy recommendations to help achieve the comprehensive development of digital inclusive finance.
